The article "IGF-1 induces the epithelial-mesenchymal transition via Stat5 in hepatocellular carcinoma" was retracted in 2024. Reasons: duplicated images; signs of a paper mill.

# IGF-1 induces the epithelial-mesenchymal transition via Stat5 in hepatocellular carcinoma

**DOI:** 10.18632/oncotarget.22952

**Published:** 2017-12-05

**Authors:** Chuanzong Zhao, Qian Wang, Ben Wang, Qi Sun, Zhaobin He, Jianguo Hong, Florian Kuehn, Enyu Liu, Zongli Zhang

**Affiliations:** ^1^ Department of General Surgery, Qilu Hospital of Shandong University, Jinan, P.R. China; ^2^ Department of Cardiology, Shandong Provincial Hospital Affiliated to Shandong University, Jinan, P.R. China; ^3^ Department of General, Thoracic, Vascular and Transplantation Surgery, University of Rostock, Rostock, Germany

**Keywords:** IGF-1, Stat5, EMT, HCC

## Abstract

It has been reported that the epithelial-mesenchymal transition (EMT) plays an important role in hepatocellular carcinoma (HCC). However, the relationship between the insulin-like growth factor-1 (IGF-1) and EMT of HCC was not fully elucidated. In the present work, we found that the expression of N-cadherin, Vimentin, Snail1, Snail2, and Twist1 was positively associated with IGF-1R expression, while E-cadherin expression was negatively associated with IGF-1 expression in human HCC samples. Furthermore, we observed that IGF-1 up-regulated the expression of N-cadherin, Vimentin, Snail1, Snail2 and Twist1, and down-regulated the expression of E-cadherin. In addition, Stat5 was induced in IGF-1-treated HepG2 and Hep3B cells, and Stat5 inhibition or siRNA significantly affected IGF-1-induced EMT in HepG2 and Hep3B cells. In conclusion, IGF-1 induces EMT of HCC via Stat5 signaling pathway. Thus, IGF-1/Stat5 can be recommended as a potential and novel therapeutic strategy for HCC patients.

## INTRODUCTION

Hepatocellular carcinoma is the leading factor in cancer-associated deaths all over the world [1–3]. Therapy outcome and prognosis for patients with HCC were demonstrated to be very poor in spite of operation combined with radiotherapy. In recent years, the 5-year overall survival rate of HCC patients accounts for nearly 15% [4]. In addition, patients suffered from different situations, iincluding resistance to chemo-radiotherapy, metastatic tendencies, and diagnosis at advanced stages, which lead to low survival rate and poor life status [5–8]. Thus, it is essential to hunt for a novel way to minimize the progression of HCC.

IGF family and their receptors play an important role in the development of tumors [9]. Recently, the role of IGF-1/IGF-1R signaling in human solid tumors has been widely reported, including lung cancer, gastric cancer [10, 11]. Recent reports have indicated that IGF-1 facilitates the progression of lung cancer by regulating cell proliferation, angiogenesis, immune evasion, and metastasis [12]. In addition, it should be noted that Stat5 was associated with IGF-1-induced angiogenesis in many types of cancers. Kalita A et al demonstrated that IGF-1 induced upregulation of cyclin D1 expression in neural cell lines via the JAK/STAT5 signaling pathway [13]. However, no studies have been reported on the role of Stat5 in IGF-1-modulated EMT of HCC.

In this study, our study aims to find the relationship between IGF-1R and EMT biomarkers (E-cadherin, N-cadherin, Vimentin, Snail1, Snail2, Twist1) in HCC samples, and then we determined the impact of IGF-1 on cell proliferation, migration and invasion of HCC cells using *in vitro* assay. Finally, we knockdown the expression of Stat5, and observed the effect of Stat5 on IGF-1-induced EMT in HepG2 and Hep3B cells. The study may provide novel insights for the treatment of HCC patients.

## RESULTS

### Expressions and correlations of IGF-1R and EMT biomarkers in human HCC tissues

It has been reported that both IGF1R and EMT were involved in the metastasis of HCC. Firstly, we investigated the relationship between the expression IGF1R and EMT biomarkers in human HCC tissues using qRT-PCR assay. Our data demonstrated that the IGF1R expression was significantly negatively associated with E-cadherin expression in HCC tissues (p=0.014) (Figure 1a). In addition, the expression of IGF-1R was significantly positively associated with the expression of N-cadherin, Vimentin, Snail1, Snail2, and Twist1 (all p<0.05) (Figure 1b-1f), which indicates that IGF-1/IGF-1R axis seems to be involved in EMT of human HCC.

**Figure 1:** Correlation between IGF-1R and EMT markers in human HCC tissues IGF1R, E-cadherin, N-cadherin, Vimentin, Snail1, Snail2, and Twist1 expression was determined in 35 human HCC tissues by qRT-PCR. Pearson correlations analysis were used to compare the mRNA expression of IGF1R and E-cadherin **(a)**, N-cadherin **(b)**, Vimentin **(c)**, Snail1 **(d)**, Snail2 **(e)**, or Twist1 **(f)** in HCC tissues. Target gene expression levels were normalized to GAPDH, and the data from three independent experiments are presented.

### Stat5 expression is induced in IGF-1-treated HepG2 and Hep3B cells

Next, we conducted western blotting to explore whether Stat5 expression is induced in IGF-1-treated HepG2 and Hep3B cells. Our results suggested that IGF-1 induced an obvious upregulation of phosphorylated Stat5 in a time and concentration-dependent manner in HepG2 cells (Figure 2a). Furthermore, IGF-1 induced an obvious upregulation of phosphorylated Stat5 in a time and concentration-dependent manner in Hep3B cells (Figure 2b). At the same time, we determined 100 ng/ml of IGF-1 for subsequent assays.

**Figure 2:** The effect of IGF-1 on Stat5 signaling in HepG2 and Hep3B cells **(a)** HepG2 cells (5×10^5^ cells/well) were treated with or without IGF-1 at 100 ng/ml for the indicated time (0, 3, 6 h) or at different concentrations (0, 50, 100 ng/ml) for 6 h. The protein levels of p-Stat5 and Stat5 were determined by western blotting. **(b)** Hep3B cells (5×10^5^ cells/well) were treated without or with 100 ng/ml IGF-1 for 6 h; p-Stat5 and Stat5 protein levels were determined by western blotting. Target gene expression levels were normalized to GAPDH, and the data from three independent experiments are presented.

### Stat5 is involved for IGF-1-induced wound closure of HepG2 and Hep3B cells

To investigate the role and mechanism of IGF-1 in the migration of HepG2 and Hep3B cells, we conducted the wound healing assays. IGF-1 obviously promoted HepG2 and Hep3B cell wound closure in a time-dependent manner (Figure 3). Moreover, it should be noted that the Stat5 inhibitor markedly prevented IGF-1-induced wound closure of HepG2 and Hep3B cells (Figure 3).

**Figure 3:** Stat5 inhibitor reduced IGF-1-induced wound closure in HepG2 and Hep3B cells HepG2 and Hep3B cells were incubated with medium alone, IGF-1, IGF-1 plus the Stat5 inhibitor or Stat5 inhibitor for 24 h (IGF-1, 100 ng/ml; inhibitor, 30 μM). Microscopic photography was performed at several time points (0, 6, 12, 24 h) after wound generation on a confluent monolayer of HepG2 and Hep3B cells (magnification, ×200). **(a)** Graphs show the wound closure of HepG2 cells in different groups at 0 h and 24 h respectively. **(b)** Graphs show the wound closure of Hep3B cells in different groups at 0 h and 24 h respectively. Data are presented as Mean ± SEM of three independent experiments. The comparisons were evaluated by Kruskal-Wallis one-way analysis of variance on ranks. ^*^p<0.05, IGF-1 compared with medium and the Stat5 inhibitor, respectively. Note: NS=normal saline.

### Stat5 is involved in IGF-1-induced migration of HepG2 and Hep3B cells

We further confirmed the metastatic properties of IGF-1-treated HepG2 and Hep3B cells using migration assays. We found that HepG2 and Hep3B cell lines exhibited stronger migratory capacity in response to IGF-1 treatment than control (Figure 4). Furthermore, the Stat5 inhibitor markedly prevented IGF-1-mediated migration of HepG2 and Hep3B cells (Figure 4).

**Figure 4:** Stat5 inhibitor impaired IGF-1-induced migration of HepG2 and Hep3B cells **(a)** Images of migratory HepG2 cells on the bottom surface of the transwell membrane (magnification, ×200). Graphs depict the number of migratory HepG2 cells. **(b)** Images of migratory Hep3B cells on the bottom surface of the transwell membrane (magnification, ×200). Graphs depict the number of migratory Hep3B cells. Data are presented as mean ± SEM of three independent experiments. The comparisons were analyzed by Kruskal-Wallis one-way analysis of variance. ^*^p<0.05, IGF-1 compared with medium and the Stat5 inhibitor, respectively. Note: NS=normal saline.

### IGF-1 induces EMT via Stat5 in HepG2 and Hep3B cells

To further investigate whether IGF-1 promotes EMT progression in HepG2 and Hep3B cells, we utilized qRT-PCR and western blotting assays to evaluate the expression of EMT biomarkers after cells were treated with or without IGF-1. Our results demonstrated that the expression of E-cadherin mRNA was down-regulated, while the mRNA expression of N-cadherin, Vimentin, Snail1, Snail2 and Twist1 were up-regulated in IGF-1-treated HepG2 and Hep3B cells compared with control (Figure 5a, 5b). Furthermore, these findings above were validated by western blotting assay (Figure 5c), indicating that IGF-1 promoted EMT of HepG2 and Hep3B cells.

**Figure 5:** Stat5 inhibitor down-regulated IGF-1-induced EMT in HepG2 and Hep3B cells HepG2 and Hep3B cells were incubated with medium alone, IGF-1, or IGF-1 plus the Stat5 inhibitor for 6 or 48 h (IGF-1, 100 ng/ml; inhibitor, 30 μM). The mRNA and protein expression levels of EMT biomarkers were determined by qRT-PCR and western blotting, respectively. **(a)** E-cadherin, N-cadherin, Vimentin, Snail1, Snail2, and Twist1 mRNA levels in HepG2 cells. **(b)** E-cadherin, N-cadherin, Vimentin, Snail1, Snail2, and Twist1 mRNA levels in Hep3B cells. **(c)** E-cadherin, N-cadherin, Vimentin, Snail1, Snail2, and Twist1 protein levels in HepG2 and Hep3B cells. Relative expression was normalized to GAPDH. Expression values were then calculated based on 2-ΔΔCt method. Data are presented as mean ± SEM of three independent experiments. The comparisons were analyzed by Kruskal-Wallis one-way analysis of variance. ^*^p<0.05, IGF-1 compared with medium and Stat5 inhibitor, respectively. Note: NS=normal saline.

Next, in order to evaluate whether Stat5 knockdown is involved into IGF-1-mediated EMT of HCC, we treated cells with a Stat5 inhibitor or Stat5 siRNA before IGF-1 stimulation. And then EMT biomarkers were analyzed by qRT-PCR assay and western blotting assays. We found the Stat5 inhibitor obviously repressed IGF-1-mediated the mRNA and protein of EMT biomarkers in HepG2 and Hep3B cells (Figure 5a, 5b). In addition, qRT-PCR and western blotting analysis demonstrated that Stat5 siRNA effectively repressed the expression of Stat5 after post-transfection 48 h (Figure 6a, 6b). We found the Stat5 siRNA also repressed IGF-1-mediated the mRNA and protein of EMT biomarkers in HepG2 and Hep3B cells (Figure 7a, 7b). All in all, these results suggested that IGF-1 induces EMT via Stat5 in HepG2 and Hep3B cells.

**Figure 6:** Stat5 knockdown by siRNA in HepG2 and Hep3B cells HepG2 and Hep3B cells (2×10^5^ cells/well) were transfected with Stat5 siRNA for 48 h, and Stat5 mRNA and protein expression was determined by qRT-PCR **(a)** and western blotting **(b)** respectively. Data were analyzed using the T test, and the results are presented as mean ± SEM of three independent experiments. ^*^p<0.05, Stat5 siRNA group compared with control.

**Figure 7:** Stat5 siRNA reversed IGF-1-induced EMT in HepG2 and Hep3B cells HepG2 (5×10^5^ cells/well) were transfected with respective siRNAs for 48 h, and then treated with IGF-1 (100 ng/ml) for additional 6 or 48 h. The mRNA and protein expression levels of EMT markers were determined by qRT-PCR and western blotting, respectively. **(a)** E-cadherin, N-cadherin, Vimentin, Snail1, Snail2, and Twist1 mRNA in HepG2 and Hep3Bs. **(b)** E-cadherin, N-cadherin, Vimentin, Snail1, Snail2, and Twist1 protein levels in HepG2 and Hep3B cells. Relative expression was normalized to GAPDH. Expression values were then calculated based on the 2-ΔΔCt method. Data were analyzed using the T test, and the results are presented as mean ± SEM of three independent experiments. ^*^p<0.05, Stat5 siRNA group compared with control.

## DISCUSSION

IGF signaling pathway modulates energy metabolism and cell growth in normal conditions. In recent years, IGF-1R and its downstream signaling activation are demonstrated to be involved in the cancer cell proliferation, anti-apoptosis and metastasis in different cancers. It has been reported that the activation of and IGF-1R downstream signaling accelerate cancer progression through an enhancement of cell proliferation, migration and invasion; however, the role of IGF-1 in EMT of HCC was not reported. Our previous studies in cancer tissues led us to further explore the effects and corresponding mechanisms of IGF-1 on EMT profiles in the development of HCC.

It has been reported that IGF-1 inhibition repressed malignant cancer cell proliferation, migration and invasion in immunodeficient mice. IGF-1 inhibition also significantly inhibited the progression of EMT, with low expression of ZEB1 and N-cadherin and high expression of E-cadherin and MITF [14]. Yao C et al demonstrated the critical roles of IGF/STAT3/NANOG/Slug signaling pathways in the progression of CRC by regulating EMT and CSCs properties [15]. Li H et al also indicates that IGF-I induced EMT by the activation of a PI3K/Akt-GSK-3β-ZEB2 signaling pathway in the development of gastric cancer [16]. In addition, emerging reports suggests that EMT progression is directly modulated by EMT transcription factors, including Snail family, Twist1, or indirectly modulated by the Stat family pathway [17–19]. Notably, we found that Stat5 was induced by IGF-1 and that Stat5 knockdown obviously inhibited IGF-1-induced HepG2 and Hep3B wound healing and migration. Therefore, our study may provide more useful information regarding the mechanism of HCC metastasis.

Based on molecular level, we further investigate whether Stat5 is also involved in IGF-1-induced EMT and found that Stat5 knockdown notably suppressed the IGF-1-induced increases in N-cadherin, Vimentin and EMT TFs expression (Snail1, Snail2, Twist1) and reversed IGF-1-mediated decrease in E-cadherin expression in HepG2 and Hep3B cells. Compared with other previous studies [20], Graham TR et al reported that IGF-I up-regulates the expression of ZEB1 in prostate cancer cells that exhibits a mesenchymal phenotype, however, ZEB1 inhibition abrogated the inhibition of E-cadherin protein, and further down-regulates the expression of N-cadherin and fibronectin proteins. As expected, ZEB1 inhibition also obviously decreases migratory and invasive potentials of prostate cancer cells than control.

In conclusion, IGF-1 signaling pathway induces EMT via Stat5 activation in HCC development. Thus, targeting of IGF-1/Stat5 or EMT may represent a novel way to decrease the development of HCC. Our work provides potential treatment strategy for HCC patients.

## MATERIALS AND METHODS

### Ethics statement

Human tissue samples used in this study were obtained with written informed consent from the patients or their relatives. This study was approved by the Ethics Committee of Qilu Hospital of Shandong University.

### Specimen collection

The study material includes 35 HCC and 35 adjacent normal tissues cases from Qilu Hospital of Shandong University, treated between 2015 and 2016. All patients underwent surgery only or postoperative adjuvant therapy. The patients’ clinicopathologic information was obtained from the pathology department archive and was confirmed by hospital medical records. All patients consent forms were obtained prior to our study. Those who had received preoperative chemotherapy, radiotherapy, and embolization will be excluded. All HCC patients were classified based on the criteria of American Joint Committee on Cancer Staging Manual, Seventh Edition (2010).

### Cell culture

The human HCC cell line HepG2 and Hep3B cell line were purchased from ATCC (Manassas, VA, USA). Cells were routinely cultured in DMEM (Invitrogen) supplemented with 5% fetal bovine serum (Sigma) at 37°C under 5% CO2. Recombinant human IGF-1 was obtained from PeproTech (Rocky Hill, NJ). STAT5 inhibitor was purchased from Calbiochem (San Diego, Calif., USA).

### Wound healing assay

HepG2 and Hep3B cells (3×10^5^ cells/well) were seeded in six-well plates and incubated overnight. After cells had reached 80-90% confluence, the culture medium was removed, and a denuded area of constant width was created by mechanical scraping with a sterile 200-μl pipette tip. Cell debris was removed, and the monolayer was washed three times with serum-free medium. The cells were cultured for an additional 24 h, and wound closure was monitored and photographed under a microscope. Results are expressed as migration indices.

### Cell migration assays

Migratory profiles were evaluated using Costar 24-well plates containing polycarbonate filter inserts with 8-mm pores. HepG2 and Hep3Bs (3×10^5^ cells/well) were added to the upper inserts and resuspended in serum-free medium. After 24 h, non-migrating cells were removed, and the underside of the insert was stained with crystal violet. Cells that had migrated into the lower chamber medium were collected and counted. Migration was calculated in terms of total cells on the lower membrane surface.

### RNA interference

The Stat5 and control siRNAs (human STAT5-siRNA, sc-29495; control-siRNA, sc-37007) were obtained from Santa Cruz Biotechnology. siRNAs were transfected into HepG2 and Hep3B cells with the siRNA Reagent System (sc-29528, Santa Cruz Biotechnology) at a final concentration of 80 nM for 48 h according to the manufacturer’s protocol.

### Quantitative real-time PCR

HepG2 and Hep3B cells (3×10^5^ cells/well) were seeded in 12-well plates and incubated overnight. For inhibitory assays, the cells were stimulated with human IGF-1 (100 ng/ml) in the presence of the Stat5 inhibitor (30 μM) or medium for an additional 6 h. For RNA interference experiments, HepG2 and Hep3B cells (1×10^5^ cells/well) were transfected with siRNA for 48 h and then treated with human IGF-1 (100 ng/ml), respectively, for an additional 6 h. Then, total RNA was extracted. Reverse transcription and real-time quantitative PCR (qRT-PCR) were performed as previously described, and the mRNA levels of target genes were normalized to those of GAPDH. The primer sequences used for PCR are presented in Table 1.

**Table 1:** Sequence of primers used for qRT-PCR amplification

Gene	Sense	Anti-sense
IGF-1R	5′-GTCGAAGAATCGCATCATCA-3′	5′-GCATCCTGCCCATCATACTC-3′
E-cadherin	5’-TTCTTCGGAGGAGAGCGG-3’	5’-CAATTTCATCGGGATTGGC-3’
N-cadherin	5’-AGAGGCAGAGACTTGCGAAAC-3’	5’-ACACTGGCAAACCTTCACGC-3’
Vimentin	5’-CAGGCAAAGCAGGAGTCCAC-3’	5’-TATTCACGAAGGTGACGAGCC-3’
Snail 1	5’-TGCCCTCAAGATGCACATCC-3’	5’-GCCGGACTCTTGGTGCTTG-3’
Snail 2	5’-AGACCCTGGTTGCTTCAAGG-3’	5’-CAGCCAGATTCCTCATGTTTGT-3’
Twist 1	5’-GGAGTCCGCAGTCTTACGAG-3’	5’-TCTGGAGGACCTGGTAGAGG-3’
GAPDH	5’-AGAAGGCTGGGGCTCAT-TTG-3’	5’-AGGGGCCATCCACAGTCTTC-3’

### Western blotting

HepG2 and Hep3B cells (1×10^6^ cells/well) were seeded in six-well plates and incubated overnight. Protein concentrations of the lysates were quantified by using the Bradford assay to ensure equal amounts of protein loaded per lane in SDS-PAGE. Cell lysates were separated by SDS-PAGE and transferred onto PVDF membranes (Millipore, Billerica, MA, USA). The membranes were blocked in 5% BSA containing 0.05% Tween-20 and probed with the appropriate primary antibodies overnight at 4°C. The membranes were washed three times for 10 min each and incubated with horseradish peroxidase-conjugated secondary antibodies for 1 h at room temperature. Membranes were then washed as above and visualized by enhanced chemiluminescence. All the antibodies were purchased from Cell Signaling Technology (CST, Beverly, MA).

### Statistic analysis

The data are presented as the mean ± SEM. T-tests for independent events were used to evaluate the significance of differences. Data in different groups were compared by Kruskal-Wallis one-way analysis of variance. Correlations were used to analyze the relationships in HCC tissues. Statistical analyses were conducted using SPSS statistical software, version 19.0 (Chicago, IL); two-tailed results with p<0.05 were regarded as significant.

## References

[1] Gao HJ, Chen YJ, Zuo D, Xiao MM, Li Y, Guo H, Zhang N, Chen RB (2015). Quantitative proteomic analysis for high-throughput screening of differential glycoproteins in hepatocellular carcinoma serum. Cancer Biol Med.

[2] Enguita-Germán M, Fortes P (2014). Targeting the insulin-like growth factor pathway in hepatocellular carcinoma. World J Hepatol.

[3] El-Ashmawy NE, El-Bahrawy HA, Shamloula MM, El-Feky OA (2014). Biochemical/metabolic changes associated with hepatocellular carcinoma development in mice. Tumour Biol.

[4] Hernández-Breijo B, Monserrat J, Román ID, González-Rodríguez Á, Fernández-Moreno MD, Lobo MV, Valverde ÁM, Gisbert JP, Guijarro LG (2013). Azathioprine desensitizes liver cancer cells to insulin-like growth factor 1 and causes apoptosis when it is combined with bafilomycin A1. Toxicol Appl Pharmacol.

[5] Weng CJ, Hsieh YH, Tsai CM, Chu YH, Ueng KC, Liu YF, Yeh YH, Su SC, Chen YC, Chen MK, Yang SF (2010). Relationship of insulin-like growth factors system gene polymorphisms with the susceptibility and pathological development of hepatocellular carcinoma. Ann Surg Oncol.

[6] Bender H, Wiesinger MY, Nordhoff C, Schoenherr C, Haan C, Ludwig S, Weiskirchen R, Kato N, Heinrich PC, Haan S (2009). Interleukin-27 displays interferon-gamma-like functions in human hepatoma cells and hepatocytes. Hepatology.

[7] Fransvea E, Mazzocca A, Antonaci S, Giannelli G (2009). Targeting transforming growth factor (TGF)-betaRI inhibits activation of beta1 integrin and blocks vascular invasion in hepatocellular carcinoma. Hepatology.

[8] Hernández-Espinosa D, Miñano A, Martínez C, Ordoñez A, Pérez-Ceballos E, de Arriba F, Mota RA, Ferrer F, González M, Vicente V, Corral J (2008). Inhibition of proteasome by bortezomib causes intracellular aggregation of hepatic serpins and increases the latent circulating form of antithrombin. Lab Invest.

[9] Yeo CD, Kim YA, Lee HY, Kim JW, Lee SH, Kim SJ, Kwon SS, Kim YH, Kim SC (2017). Inhibiting IGF-1R attenuates cell proliferation and VEGF production in IGF-1R over-expressing EGFR mutant non-small cell lung cancer cells. Exp Lung Res.

[10] Xu L, Zhou R, Yuan L, Wang S, Li X, Ma H, Zhou M, Pan C, Zhang J, Huang N, Shi M, Bin J, Liao Y (2017). IGF1/IGF1R/STAT3 signaling-inducible IFITM2 promotes gastric cancer growth and metastasis. Cancer Lett.

[11] Li C, Li J, Wu D, Han G (2016). The involvement of survivin in insulin-like growth factor 1-induced epithelial-mesenchymal transition in gastric cancer. Tumour Biol.

[12] Gan Y, Zhang Y, Buckels A, Paterson AJ, Jiang J, Clemens TL, Zhang ZY, Du K, Chang Y, Frank SJ (2013). IGF-1R modulation of acute GH-induced STAT5 signaling: role of protein tyrosine phosphatase activity. Mol Endocrinol.

[13] Kalita A, Gupta S, Singh P, Surolia A, Banerjee K (2013). IGF-1 stimulated upregulation of cyclin D1 is mediated via STAT5 signaling pathway in neuronal cells. IUBMB Life.

[14] Le Coz V, Zhu C, Devocelle A, Vazquez A, Boucheix C, Azzi S, Gallerne C, Eid P, Lecourt S, Giron-Michel J (2016). IGF-1 contributes to the expansion of melanoma-initiating cells through an epithelial-mesenchymal transition process. Oncotarget.

[15] Yao C, Su L, Shan J, Zhu C, Liu L, Liu C, Xu Y, Yang Z, Bian X, Shao J, Li J, Lai M, Shen J (2016). IGF/STAT3/NANOG/Slug signaling axis simultaneously controls epithelial-mesenchymal transition and stemness maintenance in colorectal cancer. Stem Cells.

[16] Li H, Xu L, Zhao L, Ma Y, Zhu Z, Liu Y, Qu X (2015). Insulin-like growth factor-I induces epithelial to mesenchymal transition via GSK-3β and ZEB2 in the BGC-823 gastric cancer cell line. Oncol Lett.

[17] Wu A, Chen J, Baserga R (2008). Nuclear insulin receptor substrate-1 activates promoters of cell cycle progression genes. Oncogene.

[18] Vilar L, Czepielewsk MA, Naves LA, Rollin GA, Casulari LA, Coelho CE (2007). Substantial shrinkage of adenomas cosecreting growth hormone and prolactin with use of cabergoline therapy. Endocr Pract.

[19] Fenton JI, Lavigne JA, Perkins SN, Liu H, Chandramouli GV, Shih JH, Hord NG, Hursting SD (2008). Microarray analysis reveals that leptin induces autocrine/paracrine cascades to promote survival and proliferation of colon epithelial cells in an Apc genotype-dependent fashion. Mol Carcinog.

[20] Graham TR, Zhau HE, Odero-Marah VA, Osunkoya AO, Kimbro KS, Tighiouart M, Liu T, Simons JW, O'Regan RM (2008). Insulin-like growth factor-I-dependent up-regulation of ZEB1 drives epithelial-to-mesenchymal transition in human prostate cancer cells. Cancer Res.

